The article "To Investigate the Effect of Glucocorticoids on Blood Loss during and after First Total Hip Arthroplasty and Its Safety Meta-Analysis" was retracted in 2023. Reasons: signs of a paper mill; compromised peer review; unreliable results or conclusions.

# To Investigate the Effect of Glucocorticoids on Blood Loss during and after First Total Hip Arthroplasty and Its Safety Meta-Analysis

**DOI:** 10.1155/2021/9681129

**Published:** 2021-12-17

**Authors:** Chaoqun Wang, Fulin Li, Wenhui Liu, Wenwen Huang, Qinglong Li, Dong Yin

**Affiliations:** Youjiang Medical University for Nationalities, Baise, China

## Abstract

**Objective:**

To evaluate the efficacy and safety of topical glucocorticoids for total hip arthroplasty by meta-analysis.

**Methods:**

A computerized search of the Cochrane Library, MEDLINE, EMBASE, and PubMed English databases, as well as Chinese Biomedical Literature Database, vipu Chinese Science and Technology Journal Database, Wanfang database, and Chinese Knowledge Net Database, was performed to include all randomized controlled trials (RCTs) regarding topical glucocorticoid therapy for postoperative bleeding after THA according to the inclusion criteria. The quality evaluation criteria of RCTs, as stated in the Cochrane Handbook for Systematic Reviews of Interventions 4.2.5, were adopted for evaluation, and the meta-analysis was performed using RevMan 5.3.

**Results:**

A total of 10 articles were included, including 1,112 patients: 566 in the topical glucocorticoid group and 546 in the control group. The transfusion rate was 8.43% for topical glucocorticoids and 30.05% for the control group (*P* < 0.001), and topical glucocorticoids reduced 317.89 ml total blood loss and 76.82 ml invisible blood loss, with statistically significant differences (*P* < 0.001). The amount of intraoperative blood loss was reduced by topical glucocorticoids, but the difference was not statistically significant (*P*=0.83), and the postoperative HB value was increased by topical glucocorticoids, although the difference was statistically significant (*P* < 0.001). The incidence of DVT and PE after topical glucocorticoid application (3.03%) was greater than that of the control group (2.40%), the difference was not statistically significant (*P*=0.54), and the incidence of infection after topical glucocorticoid application (3.03%) was greater than that of the control group (2.40%). The difference was not statistically significant (*P*=0.39).

**Conclusions:**

Topical glucocorticoids can reduce the transfusion rate and blood loss in THA patients without increasing their risk of thrombosis.

## 1. Introduction

Total hip arthroplasty (THA) is widely used in many hip diseases, but its blood loss tends to be large, even requiring blood transfusion. Moreover, massive blood loss adversely affects patients and aggravates the burden on multiple organs of the body [1]. In contrast, clinical transfusion may present serious potential risks such as immune reactions, HIV, HBV transmission, and intravascular hemolysis [2]. Therefore, how to reduce the bleeding caused by THA surgery has become an increasing concern and urgent problem for orthopedic surgeons. Until today, several techniques to reduce bleeding have been applied in the clinic, including the treatment of iron, the application of EPO, controlled hypotension, autologous blood reinfusion, and the use of antifibrinolytic drugs [3]. Studies in the 1990s noted that glucocorticoids could effectively reduce surgical bleeding in THA [4]. However, much literature has studied the use of glucocorticoids in THA surgery. Most believe that glucocorticoids can reduce surgical bleeding and blood transfusion in THA and do not increase the risk of DVT. However, there are reports that glucocorticoids are not effective in reducing surgical blood loss in THA. Whether glucocorticoids can effectively reduce bleeding and transfusion in THA surgery and whether they do not increase postoperative deep vein thrombosis and pulmonary embolism remain controversial. This systematic review and meta-analysis aimed to determine whether the use of glucocorticoids in THA surgery is effective in reducing blood loss and transfusion and whether it increases the risk of deep vein thrombosis, pulmonary embolism, and other complications.

## 2. Materials and Methods

### 2.1. Literature Search

Two investigators independently searched the English electronic databases, Ovid, PubMed, and ScienceDirect, and the Chinese database, Wanfang and CNKI, from January 1990 to February 2017 [5]. The English language search keywords used were ““total hip replacement””, ““total hiparthroplasty””, ““tha””, ““thr””, ““steroid””, ““glucocorticoid””, ““dexamethasone””, ““corticosteroid””, ““cortisone””, ““methylprednisono””, ““prednisone””, ““betamethasone””. The Chinese search terms were: ““total hip arthroplasty””, ““glucocorticoids””, ““dexamethasone””, ““betamethasone””, ““methylprednisolone””, ““prednisone””, ““cortisone””, ““hydrocortisone””. The search keywords were connected with the Brownian relation formula ““and”” ““or ““or””. References from conference proceedings and related reviews were hand searched to retrospectively analyze key orthopedic meetings since 1980 and consult relevant experts in the field. Relevant literature regarding this study in the Chinese Journal of Orthopedics [6], Chinese Journal of Trauma Orthopedics [7], Chinese Journal of Trauma [8], and Chinese Journal of Bone and Joint Loss [9] was manually searched. Two investigators independently retrieved relevant literature for screening, and by reading the title of the literature as well as abstracts to remove the literature, the reviewer could not request the full text for full-text reading.

### 2.2. Inclusion and Exclusion Criteria

Inclusion criteria are as follows: (1) types of studies: clinical randomized controlled trials (RCTs); (2) subjects: initial unilateral total hip arthroplasty with consistent baseline levels in both groups (demographic factors such as gender and age); ③ the test group received glucocorticoids intravenously or orally before, during, or after surgery; and (4) the evaluation indicators included the following: transfusion rate, invisible blood loss, postoperative drainage volume, total postoperative blood loss, hemoglobin (HB) drop value, Hb value at 24 h postoperation, incidence of postoperative deep vein thrombosis (DVT) and pulmonary embolism (PE), and incidence of wound infection.

Exclusion criteria are as follows: (1) nonrandomized controlled trials; (2) the patients studied were unicondylar replacement, hip arthroscopy, and hip revision; (4) studies with the above evaluation indicators were not included; (5) excluding literature published in the same duplicate (6); excluded reviews, meta-analyses, and reviews where data could not be extracted.

### 2.3. Quality Assessment of Included Literatures [10]

The methodological quality assessment of the included studies was performed using the criteria for the quality assessment of RCTs in (Cochrane Handbook for Systematic Reviews of Interventions 4. 2. 5): (1) whether the random method selection was correct; (2) whether or not blinding was employed and was the choice of blinding correct; (3) whether allocation concealment; (4) with or without loss to follow-up or withdrawal and with or without loss to follow-up or withdrawal in an intention to treat analysis; and (5) whether the baseline was consistent. A literature review was conducted on the selection of randomized methods, whether blinding was used at the time of randomization, with or without loss to follow-up, or withdrawal.

### 2.4. Evaluation Index Extraction and Statistical Analysis

A table was developed to extract evaluation indicators, and two investigators extracted data from the literature in accordance with the table content. RevMan 5.3 software was used for statistical analysis. The amount of postoperative drainage, total blood loss, invisible blood loss, intraoperative blood loss, 24 h postoperative HB value, and Hb reduction using topical glucocorticoids were expressed as weighted mean difference (WMD) with 95% confidence interval (CI). The incidence of blood transfusion, incidence of DVT and PE, and incidence of infection were expressed using relative risk (RR) with 95% CI. Heterogeneity between studies was tested using the *I*^2^ and *X*^2^ tests, and if *P* > 0.1 or *I*^2^ ≤ 50%, there was no significant heterogeneity, data were pooled using a fixed-effects model (Mantel–Haenszel method, Multiple studies were considered significant if *P* < 0.1 or *I*^2^ > 50%.

There was heterogeneity among the results, the source of heterogeneity was analyzed, subgroup analysis was performed for those with heterogeneity, when heterogeneity could not be eliminated and clinical consistency was present, and the data were pooled by using random effects model (inverse variant method) [11].

## 3. Results

### 3.1. Quantity and Quality Assessment of Retrieved Literature

After the search, 290 articles were identified: 115 in English and 175 in Chinese. After removing duplicates by endnote software, a total of 120 pieces of literature were screened. Sixty-five articles were excluded by reading the title and abstract of the articles, and the remaining by reading the full text, resulting in a total of 10 RCTs after exclusion [12–21]. A total of 1,112 patients were included: 566 in the topical glucocorticoid group and 546 in the control group. The pieces of literature were all published until 2013, the average age of patients was 50.00–76.90 years, the application dose of glucocorticoids was 1–3 g, the application mode was mainly through drainage tube injection [18, 21] and intraoperative infiltration of glucocorticoids [13, 15, 19], the other was joint cavity injection [12, 17, 20], 2 studies did not use drainage tubes [12, 17], 1 study did not mention whether a drain was used or not [12], the rest of the studies used a drain, and the patients' general conditions are shown in Table 1.

All studies clearly described the random sequence generation method and the method of allocation concealment. Except for Yuan Xiaowei's study [21], all other studies clearly described the blinding of participants and data statistics. In contrast, incomplete outcome data were clearly described in other studies, except for the study by Yue [15]. For publication bias and other bias, there is less literature that accurately describes it. A detailed description of the included literature quality reviews is presented in Table 2.

### 3.2. Comparison of the Efficacy of Topical versus Intravenous Glucocorticoids

#### 3.2.1. Transfusion Rate

Eight publications analyzed transfusion rates in both cohorts without statistical heterogeneity between studies (*x*^2^ = 2.27, *I*^2^ = 0%, *P*=0.95), using a fixed effects model. Topical glucocorticoid use was associated with a reduced transfusion rate of 8.43% compared with 30.05% in the control group (RR = 0.28, 95% CI: 0.20–0.39, *P* < 0.001); see Figure 1.

#### 3.2.2. Total Blood Loss, Hidden Blood Loss, and Intraoperative Blood Loss

Seven papers analyzed postoperative THA blood loss with statistical heterogeneity between studies (*x*^2^ = −20.87, *I*^2^ = 71%, *P*=0.002) using a random effects model, topical glucocorticoids were found to reduce total blood loss by 317.89 ml compared to controls with a statistically significant difference (WMD = −317.89, 95% CI: −377.67 to −258.12, *P* < 0.001). Invisible blood loss was analyzed in 1 study, and topical glucocorticoid application reduced the amount of invisible blood loss by 76.82 ml, which was statistically significant (WMD = −76.82, 95% CI: −89.77 to −63.87, *P* < 0.001). Intraoperative blood loss was analyzed in 3 publications, and the reduction of intraoperative blood loss by topical glucocorticoids was not statistically significant (WMD = −1.18, 95% CI: −12.10–9.74, *P*=0.83); see Figure 2.

#### 3.2.3. Drainage Volume

The amount of drainage after THA was analyzed in six articles, with significant statistical heterogeneity between studies (*x*^2^ = 3106.36, *I*^2^ = 93%, *P* < 0.001), using a random effects model, topical glucocorticoid application was found to reduce the drainage volume of 140.21 ml when compared with the control group, with a statistically significant difference (WMD = −140.21, 95% CI: −189.19 to −91.22, *P* < 0.001); see Figure 3.

#### 3.2.4. The HB Value 24 h after Operation as well as the HB Drop Value

Five pieces of literature analyzed the HB value at 24 h after operation without statistical heterogeneity among studies (*x*^2^ = 4.09, *I*^2^ = 2%, *P*=0.39). Using the fixed effect model, topical glucocorticoids could increase the postoperative HB value, and the difference was statistical.

Significance (WMD = 9.18, 95% CI: −7.32–11.05, *P* < 0.001): two articles reported the value of HB decline after surgery, and topical glucocorticoids could reduce the value of HB decline with a significant difference (WMD = −13.40, 95% CI: −15.99–10.81, *P* < 0.001); see Figure 4.

#### 3.2.5. Comparison of Incidence of DVT and PE Postoperative Infection

The incidence of postoperative DVT and PE was analyzed in eight articles, with no statistical heterogeneity between studies (*x*^2^ = 1.12, *I*^2^ = 0%, *P*=0.89), using a fixed effects model, the incidence of DVT and PE after topical glucocorticoid application (3.03%) was greater than that of the control group (2.40%), and the difference was not statistically significant (RR = 1.27, 95% CI: 0.59–2.74, *P*=0.54); see Figure 5. Four articles analyzed the rate of postoperative infection in two groups of patients, the incidence of postoperative infection after topical application of glucocorticoids (3.03%) was greater than that in the control group (2.40%), and the difference was not statistically significant (RR = 2.30, 95% CI: 0.34 to 15.38, *P*=0.39); see Figure 5.

#### 3.2.6. Hip Function Score

Three studies analyzed the postoperative hip functional score, two studies analyzed the Harris score [22], and one study analyzed the Oxford hip functional score (OHS). For Harris score, topical glucocorticoids could enhance hip function, and the difference was statistically significant (WMD = 1.12, 95% CI: 0.39–1.84, *P*=0.003). For OHS, there was no significant difference in the effect of topical glucocorticoids compared with the control group (WMD = −2.80, 95% CI: −7.04–1.44, *P*=0.20); see Figure 6.

#### 3.2.7. Subgroup Analysis

Because of significant heterogeneity in total blood loss and drainage volume, studies with general data found inconsistency in the doses of topically applied glucocorticoids, analyzed according to total doses of 1 g, 2 g, and 3 G, with 3 publications included at a total dose of 1 g [15, 18, 20], with statistical heterogeneity between studies (*x*^2^ = 7.05, *I*^2^ = 72%, *P*=0.03). Topical application of glucocorticoids reduced 367.71. At a total dose of 3 G [12, 14], there was no statistical heterogeneity between studies (*x*^2^ = −1.52, *I*^2^ = 34%, *P*=0.22), and topical glucocorticoids reduced 358.28 ml total blood loss with a statistically significant difference (WMD = −358.28, 95% CI: −26 to −286.31, *P* < 0.001).

## 4. Discussion

Accelerated recovery after surgery (ERAS) refers to the provision of highly efficient and high-quality medical services after a series of simple and effective perioperative management measures that reduce surgical, traumatic stress reaction and postoperative complications, alleviate patient suffering, and shorten hospital stay [23, 24]. Numerous studies have confirmed that eras are effective in reducing postoperative complications of joint arthroplasty, reducing the length of hospital stay, and improving patient satisfaction [25]. Moreover, one of the key points of eras application in joint arthroplasty is to reduce postoperative stress and inflammation [26].

The inflammatory response is one of the important mechanisms underlying the stress response after surgical trauma. It is closely related to postoperative pain, postoperative nausea and vomiting (PONV), fatigue, muscle strength loss, sleep disturbance, and so on. Therefore, alleviating the postoperative inflammatory response can help reduce postoperative complications, shorten hospital stay, and achieve the goal of accelerating rehabilitation after joint replacement [27]. Glucocorticoids, as a commonly used and effective agent to inhibit inflammatory responses, have been widely used in various types of surgery and are proven to have good effects [28, 29]. In recent years, domestic and foreign scholars have conducted relevant studies on the systemic application of glucocorticoids in TKA, but high-quality, relevant studies were few, the level of evidence was low, and the results were still controversial [30]. It is believed that systemic administration of glucocorticoids can effectively relieve pain, reduce PONV symptoms, and accelerate recovery in the perioperative period of total knee arthroplasty (TKA) after TKA [31]. There have also been studies with reservations regarding the efficacy of systemic glucocorticoid use in TKA [32].

THA has become a more mature surgical technique in the clinic. However, it is a traumatic treatment, and postoperative fever, infection, deep vein thrombosis, prosthesis loosening, fracture, dislocation, limb malalignment, and heterotopic ossification often occur, especially with fever, infection, and deep vein thrombosis [33]. In the early postoperative period, appropriate rehabilitation training is necessary to promote venous return of the affected limb, reduce swelling, prevent deep vein thrombosis of the lower extremity, reduce adhesion to surrounding tissues, increase the strength of surrounding muscle groups, enhance joint stability and the weight-bearing capacity of bone, shorten rehabilitation time, and improve the functional status and quality of life of the limbs. Reducing the incidence of various types of complications and so on has a very important role [34]. However, patients often experience pain affecting normal rest, sleep, and diet, which can affect wound healing and postoperative functional exercises, severely affecting hip functional recovery and patient satisfaction [35]. Currently, adjuvant therapy with glucocorticoids (GC) is applied to patients undergoing surgical procedures clinically, in the perioperative period to reduce pain and reduce complications [36].

GC has many physiological and pharmacological effects, which mainly include the following: (1) obviously suppressing the inflammatory response induced by various factors, inhibiting the movement of inflammatory cells to the site of inflammation, stabilizing the lysosomal membrane, reducing serotonin and IL-1*β*, releasing inflammatory mediators such as IL-6, TNF-a, and bradykinin, thereby alleviating symptoms such as redness, heat, and pain [37]; (2) moderating the body's response to endotoxin, inhibiting the hypothalamic response to pyrogens, inhibiting the production and release of leukocyte pyrogens, decreasing the sensitivity of thermoregulatory centers to pyrogens, and having an antipyretic effect on hyperthermia [38]; (3) antishock effect and the effect of increasing the body's stress capacity; and (4) inhibiting the proliferation of fibroblasts, reducing the production of collagen fibers, and so on.

The results of the meta-analysis showed that topical glucocorticoids, which reduced the blood transfusion rate, total blood loss, and invisible blood loss; increased postoperative Hb; decreased HB drop values; and enhanced hip function, did not increase the incidence of postoperative DVT, the incidence of wound infection, or the OHS score and were not statistically significant for intraoperative blood loss. THA is associated with significant blood loss due to procedures such as intraoperative muscle transection plus reaming, which can cause significant overt blood loss. On the contrary, invisible blood loss is the focus of attention among orthopedic surgeons in recent years, with studies indicating that invisible blood loss accounts for 60% of total blood loss, and the mechanism responsible for invisible blood loss may have hemolysis caused by intraoperative RBC rupture. The interstitial exudation doctrine [39], with studies suggesting a fibrinolytic activation period after 24 h of surgery, further increases postoperative blood loss [40]. Glucocorticoids, as a commonly used and effective agent to inhibit inflammatory responses, have been widely used in various types of surgery and are proven to have good effects [41]. Although glucocorticoids theoretically do not increase the amount of fibrin, Li et al. [42, 43] suggested that intravenous glucocorticoids inhibit fibrinolysis throughout the body, combined with the fact that hip replacement patients, who are mostly elderly patients, would increase the incidence of postoperative DVT and PE. Topical application of glucocorticoids concentrates glucocorticoid drug concentrations around the joint cavity via various routes [44]. In this study, the transfusion rate of topical glucocorticoids was 8.43% compared with 30.05% in the control group (RR = 0.28, 95% CI: 0.20–0.39, *P* < 0.001), although Wang [45] concluded by meta-analysis of randomized controlled trials and retrospective comparative studies that topical glucocorticoid administration could reduce the transfusion rate without increasing the rates of DVT and PE. However, the Chinese databases were not searched, and only 4 RCTs were included, which did not compare invisible blood loss and postoperative hip function scores.

The strengths of this study are that only RCTs were included; non-RCTs were excluded; and invisible blood loss, 24 h postoperative HB value, and hip function score were compared, which strengthened the evidence grade and further demonstrated that topical glucocorticoids could reduce perioperative total blood loss and invisible blood loss, increase postoperative HB value, and enhance the Harris score in hips.

Postoperative DVT and PE are more dangerous postoperative complications, which threaten the life safety of patients once they form a PE [46]. The results of the eight included articles showed no significant difference in the incidence of DVT and PE after topical glucocorticoids, which suggests that topical glucocorticoids do not increase the incidence of postoperative thrombus while reducing postoperative blood loss. Nevertheless, the results were consistent in the study of [47], which compared seven series of hip replacement patients with topical glucocorticoids. Topical glucocorticoids can reduce postoperative blood loss without increasing the chance of postoperative thrombosis in patients with total hip replacement. Compared with the intravenous application of glucocorticoids, the topical application of glucocorticoids can reduce the systemic blood concentration and avoid the occurrence of thrombus [48]. In conclusion, topical glucocorticoids can reduce postoperative blood loss and reduce the rate of blood transfusion without increasing postoperative thrombosis in THA patients. However, because various studies used different doses and different methods of topical application, the direction of future research should focus on the optimal dose of glucocorticoids and the efficacy of topical glucocorticoids compared with intravenous glucocorticoids to explore the most applicable volume and optimal application route.

Although long-term administration of glucocorticoids has an increased risk of infection, gastrointestinal bleeding, and so on, short perioperative glucocorticoid administration is not associated with such risks [49]. A meta-analysis involving 71 studies confirmed that short perioperative glucocorticoid administration does not increase the risk of postoperative complications in patients [50]. Currently, although relevant studies on the systemic application of glucocorticoids in THA all agree that the glucocorticoid group has the same postoperative complication rate as the control group, some studies have found that local application of glucocorticoids in the hip joint cavity may increase the risk of postoperative infection [51]. Therefore, we still need to pay more attention before definitive conclusions can be drawn.

This study mainly has 3 deficiencies: (1) the included literature has a small sample size, which is difficult to cause bias to the results and generates uncertain conclusions [52]; (2) because the statistical results of some indicators such as hip function and thrombotic markers were few, a meta-analysis could not be performed and only descriptive statistics could be performed; and (3) the limited number of included studies in the literature was insufficient to perform subgroup analyses targeting high or low glucocorticoid doses. However, this systematic review and meta-analysis is the first to synthesize the relevant, high-quality literature to date, perform a normative meta-analysis according to PRISMA principles and processes, and comprehensively analyze the use value of systemic glucocorticoids in THA accelerated rehabilitation. We believe that the results of this study will be an important guiding value for clinical work [53].

The results of the present study suggest that topical glucocorticoids can reduce the transfusion rate and blood loss in THA patients without increasing their risk of thrombosis.

## Figures and Tables

**Figure 1:** Comparison of transfusion rates between the two groups.

**Figure 2:** Comparison of total and invisible postoperative blood loss as well as intraoperative blood loss between the two groups.

**Figure 3:** Comparison of postoperative drainage volume between two groups.

**Figure 4:** Comparison of Hb values and Hb decline at 24 h after operation between the two groups.

**Figure 5:** Comparison of the incidence of postoperative DVT as well as PE between the two groups.

**Figure 6:** Comparison of postoperative hip function scores between the two groups.

**Table 1:** General condition of included study patients.

Investigators and years	T/C (people)	Mean age (years) (T/C)	Intervene	Drainage tube	Transfusion criteria	Prosthesis type
Martin [12]	25/25	62.96/63.92	100 mg hydrocortisone, 2 h before operation and push still + 8 h after the second dose	Not used	Hb ＜ 7	NS
Wei [13]	102/100	60.2/63.9	10 mg dexamethasone, 1 h preoperative static push + second dose during surgery	They were opened after 30 min of clipping and removed 24 h after surgery	Hb ＜ 9	Cementless prostheses
Alshryda [14]	80/81	66/63	100 mg hydrocortisone, 2 h before operation push + 8 h after second dose + 8 h after third dose	NS	NS	NS
Yue [15]	52/49	60.9/63.7	8 mg or 16 mg dexamethasone at the end of surgery and pushed to rest	They were opened after 30 min of clipping and removed 24 h after surgery	Hb ＜ 7	Cementless prostheses
Jiajing Ye [16]	40/40	71.5/71.3	With 125 mg methylprednisolone, i.p.	They were opened 3 h after clipping and removed 24 h after surgery	Hb ＜ 7.5	Cementless prostheses
Ding, min [17]	30/30	60.00/61.00	100 mg hydrocortisone, 2 h before operation push + 8 h after second dose + 8 h after third dose	Not used	Hb ＜ 8	DePuy joints
Yin Han [18]	30/30	50.00/53.56	100 mg dexamethasone, and pushed statically before anesthesia	They were opened after 6 h of clipping and removed at 48 h after surgery	Hb ＜ 7	Biotype prosthesis
Yan, Liang [19]	107/107	54.10/62.23	10 mg dexamethasone, i.p.	Not used	Hb ＜ 7	Cementless prostheses
Fanfucheng [20]	56/44	66.04/66.50	100 mg hydrocortisone, 2 h before operation and push still + 8 h after the second dose	They were opened after 2 h of clipping and removed 24 h after surgery	Hb ＜ 7	Cementless prostheses
Yuan, Xiaowei [21]	40/40	76.90/76.86	10 mg dexamethasone, 1 h preoperative static push + second dose during surgery	The interval was 1 h and was removed 48 h after surgery. They were removed 48 h after surgery	Hb ＜ 9	DePuy total hip instrumentation

T: glucocorticoid application, C: control group, NS: not mentioned, Hb: hemoglobin.

**Table 2:** Quality assessment of the included literature.

Investigators and years	Random sequence	Allocation concealment	Trialists and participants double-blind	Outcome assessment double-blind	Incomplete outcome data	Publication bias	Other biases
Martin [12]	Yes	Yes	Yes	Yes	Yes	Yes	Unclear
Wei [13]	Yes	Yes	Yes	Yes	Yes	Unclear	Unclear
Alshryda [14]	Yes	Yes	Yes	Yes	Yes	Yes	Unclear
Yue [15]	Yes	Yes	Yes	Unclear	Unclear	Unclear	Unclear
Jiajing Ye [16]	Yes	Yes	Yes	Yes	Yes	Yes	Unclear
Ding, min [17]	Yes	Yes	Yes	Unclear	Yes	Unclear	Unclear
Yin Han [18]	Yes	Yes	Yes	Yes	Yes	Unclear	Unclear
Yan, Liang [19]	Yes	Yes	Yes	Unclear	Yes	Unclear	Unclear
Fanfucheng [20]	Yes	Yes	Yes	Yes	Yes	Unclear	Unclear
Yuan, Xiaowei [21]	Yes	Yes	Unclear	Unclear	Yes	Unclear	Unclear

## Data Availability

The original data could be obtained from the corresponding author.
